The article "The axiological foundations of innovation in STEM education – A systematic review and ethical meta-analysis" was published in 2024. Journal: Heliyon.

# The axiological foundations of innovation in STEM education – A systematic review and ethical meta-analysis

**DOI:** 10.1016/j.heliyon.2024.e32381

**Published:** 2024-06-04

**Authors:** Fernand Vedrenne-Gutiérrez, Carolina del Carmen López-Suero, Adalberto De Hoyos-Bermea, Lorena Patricia Mora-Flores, Daniela Monroy-Fraustro, María Fernanda Orozco-Castillo, José Francisco Martínez-Velasco, Myriam M. Altamirano-Bustamante

**Affiliations:** a Grupo Transfuncional en Bioética Del Centro Médico Nacional Siglo XXI, IMSS., Av. Cuauhtémoc 330, Doctores, Mexico City, 06720, Mexico; b Departamento de Ingeniería Química, Industrial y de Alimentos, Universidad Iberoamericana, Prol. P.° de la Reforma 880, Santa Fe, 01219, Mexico City, Mexico; c Centro de Investigaciones Económicas, Administrativas y Sociales (CIECAS), Instituto Politécnico Nacional, Lauro Aguirre 120, Mexico City, 11360, Mexico; d Escuela de Ciencias de la Salud, Universidad Anahuac, Av. Universidad Anahuac 46, Huixquilucan, 52786, Estado de México, Mexico; e Departamento de Salud, Universidad Iberoamericana, Prol. P.° de la Reforma 880, Santa Fe, 01219, Mexico City, Mexico; f ESDAI - Universidad Panamericana Ciudad de México, Cda. Augusto Rodin No. 498, Insurgentes Mixcoac, Benito Juárez, 03920 Ciudad de México, CDMX, Mexico; g Facultad de Ingeniería - Universidad Panamericana Ciudad de México Cda. Augusto Rodin No. 498, Insurgentes Mixcoac, Benito Juárez, 03920 Ciudad de México, CDMX, Mexico

## Abstract

**Introduction:**

Values are crucial in decision-making, including processes related to science and technology, despite scientists often being unaware of them. Because a goal of science, technology, engineering, and mathematics (STEM) is to foster innovation, values have become fundamental in directing science and technology policies and shaping organizational cultures to leverage innovation. However, most research on STEM education has focused on improving performance or access to STEM education while overlooking its axiological configuration. This study analyzes the different value systems emerging in the current literature on STEM higher education and identifies the relevant stakeholders.

**Method:**

In this systematic review and ethical meta-analysis, we aimed to assess the most prominent studies on STEM education and its core values. We followed a Ricoeur-inspired hermeneutical methodology using Atlas ti 8.4.4. Values are identified and classified using a systematic approach to integrate axiological landscapes.

**Results:**

The literature does not explicitly discuss the value of STEM education for innovation. However, social values appear to be at the intersection and the cornerstone of basic, economic, aesthetic, and epistemic values, as most social values also manifest these four systems. The most common manifestation of the value system is the capability approach to justice, followed by the beauty of recognition and success and, in third place, racism and social disparities. The analyzed literature emphasizes STEM education's social, political, and economic determinants. However, there is an epistemic gap in the indispensable value of innovating and assessing STEM education.

**Conclusions:**

We propose an organizational culture model for STEM education that considers the goals, ends, values, and behaviors of students, teachers, educational institutions, and the government. This model can help fill the axiological gaps in STEM education.

## Highlights

• Literature on STEM education focuses on social values with a particular interest in the capability approach to justice.
• The main ethical approach to STEM education is the utilitarian. Other ethical approaches require more development.
• There are four stakeholders in STEM education: students, professors, institutions, and government.

## 1 Introduction

Modern education literature frequently uses the term science, technology, engineering, and mathematics (STEM) education. Nevertheless, there is no consensus on what this means. This lack of a clear definition has led to confusion in the field [1,2]. Traditionally, STEM education has been defined in two ways: 1) education in any individual STEM discipline and 2) education that seeks to integrate all STEM disciplines [2]. The first definition treats each science as separate from technological developments, whereas the second emphasizes a collaborative model in which science and technology are integrated. In this study, STEM education is defined as developing competencies in science, technology, engineering, or mathematics, with or without the intentional integration of separate disciplines. The distinction between scientific disciplines is more practical than an epistemological classification.

Most studies on STEM education have focused on its contents and benefits, neglecting the values that emerge in these disciplines. STEM disciplines pursue specific goals, and scientists are continuously challenged by difficult choices that interact with the social, economic, political, or ecological aspects of human existence. Given the social, political, and economic nature of STEM disciplines [3], they function as a result of interacting and competing values (axiological networks) [[4], [5], [6]]. Scientists, like all professionals, make decisions daily [7]. According to Pirozelli [7], the idea of an ethically neutral STEM can be seen in Kuhn's work on rationality. Accordingly, values permit an evaluation of something as desirable or undesirable. Even if STEM practitioners are unaware of this distinction, they use clusters of values in their practice. These values do not emerge in isolation but rather as a system [3,7].

Values are used to define something as good or desirable. Hartmann stated that these are intangible ideal entities that guide every human action. These entities can be grouped into systems [8]. According to Mounier, freedom implies adhering to a set of values to take action in one domain (and stop acting in another) [9]. Echeverría [4] states that a dozen value systems exist in technoscience. These systems also apply to broader STEM practices. Other authors have proposed different systems [6], but Echeverría offers an integral perspective that can be applied practically. This axiological pluralism stems from the idea that STEM disciplines are multidimensional and may not be reduced to epistemic matter. These proposed systems are basic, epistemic, technical, economic, military, religious, political, social, aesthetic, juridical, moral, and ecological. A thorough description of these value systems can be found elsewhere [3,4].

According to our preferred definition, it is essential to outline the relevant historical aspects to better understand STEM education's value systems. STEM education may have resulted from the technoscientific revolution (TSR) around World War II (WWII). The TSR resulted from the appearance of the so-called Big Science paradigm: a new system in which scientific activity underwent significant restructuring. Big Science is characterized by human resource specialization, extensive funding, political involvement, bureaucratization, the militarization of physics and math, and close interaction between scientists, engineers, technicians, military officers, and other professionals [3]. This new method of producing knowledge is called technoscience. The term technoscience depicts a shift in values, in which knowledge transforms from being the primary objective to a means to an end. These changes transformed how science was performed, how technology developed, and how social, political, and military characteristics were acquired [3]. Today, technoscience has been subsumed by the term STEM. As a result, STEM education has inherited some value systems from the Big Science paradigm but may also have developed different value systems according to contextual and historical factors. It is currently unknown how these value systems affect the teaching of STEM disciplines under different scenarios.

Recognizing the ethical framework and the most prominent value systems of STEM education is essential because STEM literacy is rapidly becoming required in workplaces. Thus, STEM education is of prime importance in the current curriculum at all levels [[10], [11], [12], [13], [14]]. However, STEM programs in higher education tend to have high dropout rates [14,15], the causes of which are manifold [16]. Some studies have attributed this to performance anxiety [10,16], the development of a scientific identity [13,14,17], the sacrifices that a STEM career may imply [12], and marginalization [[12], [13], [14],^18^,^19^]. Xie et al. [2] classified the determinants of education into contextual, family, and personal factors. Furthermore, STEM courses are considered intellectually inaccessible disciplines, reserved for only a few people [11,20].

As mentioned above, STEM competencies are increasingly becoming workplace assets. Consequently, STEM education is seen as one of the pillars of innovation, trampolining basic research that can later be translated into new inventions and entrepreneurship. If applied promptly, science, technology, and innovation (STI) policies can strengthen innovation systems and promote social wealth, wellbeing and economic development. Late policies come at the cost of opportunities [21].

Governments seeking to leverage STI policies must explicitly include STEM education to plant seeds for future innovation and have readily available scientific capital. STI policy is a costly investment that may not be considered a priority in some regions. Regional priorities are established by local value hierarchies. The literature has identified two types of STI cultures with their corresponding values: first movers and late-stage developers. First movers must invest considerable money in research and development and push past the *status quo*, while late-stage developers must base their work on first movers without gaining any prestige or recognition that will attract future investment and without being able to break current paradigms [21]. If they value direct action toward a culture of innovation, governments will view investments in STI policies as goods.

Culture plays a vital role in establishing value hierarchies for innovation. Certain cultures favor change and novelty, whereas others value the *status quo*. Societies can be divided into organizations with their own cultures. A broad culture permeates the organizational culture and evolves as if it were an individual with value. Organizational values are functions of the individual values of each actor within an organization, which are in constant competition. The values that persist define the culture. According to this competing value model, organizational culture has two dimensions: internal vs. external focus and flexibility/discretion vs. stability/control. Adhocracy is a culture with high flexibility and an external focus. Cultures that value stability with an external focus are market-driven. Internally focused cultures that value flexibility are clan- or family-oriented, whereas those that value control and stability are hierarchical [22]. STEM education is a culture characterized by the competing values of each actor.

Much of the research examining the determinants of STEM education attrition in higher education does so from a purely behavioral framework without considering the axiological landscape. Thus, we decided to study the value systems in the most recent literature on STEM education to point out the leading topics of discussion and research and set the agenda on topics that require further analysis. This article's research question is “What value systems emerge (axiological landscape) in current research papers on STEM higher education?” This study identifies the main actors in STEM education and proposes a model that outlines each party's responsibilities. The model harnesses innovation from course instructors and students by fostering values and virtuous scientific practices in the classroom, ultimately becoming organizational cultures seeking to solve problems through innovation.

Emphasizing values in STEM education can deepen understanding of the social and ethical implications of technoscientific innovation. Making values explicit allows teachers, parents, institutions, and governments to encourage students to immerse themselves in the ethical implications of science and promote a responsible and integral type of STEM. Furthermore, this can help incorporate cultural perspectives and ethical frameworks into STEM education, facilitating its translation into inclusive, diverse, and socially responsible disciplines. However, this requires further investigation. Dealing with abstract concepts such as values can be an epistemic challenge for many, potentially setting the stage for further complicating the already difficult job of teaching diverse students. Moreover, it may be difficult to determine which values should be prioritized and to reach a consensus on the moral good these values should point to.

## 2 Materials and methods

This systematic review followed the Participant-Intervention-Outcome (PIO) method to answer, “What are the values and attitudes toward science, technology, and innovation of undergraduate students and teachers?”. A summary of the methodological roadmap is shown in Fig. 1.

**Fig. 1:** Methodology roadmap: Different steps followed to answer the research question. In the analysis step, the hermeneutical approach lead to a deeper understanding of the axiological horizon of the narratives of the selected articles, and therefore was a key step in the ethical meta-analysis.

Fig. 2 shows the decision tree for the PIO approach. All articles related to the clinical sciences were excluded. The resulting search query was searched in three databases: Web of Science [23], Scopus [24], and PubMed [25]. These databases were selected based on their position in different regions of the world and the breadth and scope of the journal collections they cover. Only articles published in English in the past five years were included.

**Fig. 2:** Article screening decision tree that follows the PIO approach.

A manual search was conducted to identify articles on capability approaches to justice in STEM education. Duplicates were removed, and article titles were screened for relevance to the research question. The abstract, materials, and methods were thoroughly assessed. The inclusion criteria were observational quantitative, qualitative, or mixed studies; undergraduate students or teachers who participated in STEM track programs; and evaluations of attitudes, values, or determinants of success. This study analyzed the values that emerged in higher education STEM courses at baseline and without intervention.

Therefore, studies on graduate, high school, middle school, or elementary school students and interventional studies, validation studies, reviews, or studies on non-STEM track programs were excluded. The quality of the remaining studies was assessed using previously validated instruments. Quantitative studies were assessed by "Strengthening the Reporting of Observational Studies in Epidemiology (STROBE)” instrument. The “Consolidated Criteria for Reporting Qualitative Research” (COREQ) instrument was used for qualitative studies. The case studies were evaluated using the checklist proposed by Wiley [26]. Finally, mixed method studies used the “Mixed Methods Appraisal Tool” (MMAT). Only studies that scored 70 % or higher in the final assessment were included to obtain the best articles. The details of each instrument's items, validity, and reliability are described elsewhere. All the instruments mentioned above are checklists detailing the robustness of each study design. Experts have developed and validated such checklists [[27], [28], [29]].

After quality assessment, only studies scoring more than 70 % were included in the final analysis. The articles received 1, 0.5, or 0 for each item. The total score was calculated by adding each item and dividing by the total number of items. Given the various educational research methodologies, these instruments identify articles with a standard study design and the information required to perform an axiological meta-analysis. Articles that scored under 70 % were not excluded due to poor quality but rather because their research design could not be categorized in the analytical framework used for the present study.

A meta-analysis is a mixed-method analysis of data from different sources encompassing quantitative and qualitative approaches. The operational definition of an ethical meta-analysis involves systematically gathering similar studies that answer a particular research question to identify emerging values and interests within the narrative. Hermeneutic analysis was conducted for each selected article using Ricoeur's method [30].

Hermeneutic analysis helps identify and describe emerging values and interests expressed in symbols or metaphors within a specific narrative and interprets them in the context in which they emerge. This method was performed in three stages: 1) naïve reading, 2) in-depth analysis and coding, and 3) final interpretation, as shown in Fig. 1. This methodology helps answer our research questions, as it allows for identifying abstract content that may not be explicit throughout the literature. Values do not always emerge explicitly and are often reflected in authors’ interpretations of different situations. Analyzing the literature results in a traditional systematic review, which would miss the interpretation of symbols and metaphors within the narrative that allows us to identify value systems.

Two authors created a codebook based on Echeverria's model, one of the few value system models developed for application. A code is a tag that summarizes an emerging topic or value. Codes are grouped into families and value systems. Descriptions of each system are presented in Table 1. Definitions were discussed and agreed upon, depending on their applicability to teaching STEM [3]. Each coder proceeded to code a section of one article independently using Atlas. ti, version 8.4.4. This process included a naïve reading of the selected section and a second thorough review in which value systems were assigned to sections in the text that manifested a particular value system.

**Table 1:** Value systems and their meaning.

System	Interpretation
Basic Values:	Those related to respect for human and animal life and dignity
Juridical Values:	Related to the application of justice and regulations
Ecological Values:	Related to the respect of the world and the environment
Social Values:	Related to the social benefits brought by STEM. It may include social prestige, social improvement, sense of belonging, or social wellbeing … Non-limitative examples may include identity, belonging, team-building.
Moral Values:	These values help deciding what is good from what is wrong.
Epistemic Values:	These values are related to the building of knowledge, they may include correctness, mastery, simplicity …
Political Values:	They include those values related to the building of governance and the public space.
Economic Values:	Related to exchange of needs. They relate to transactions, whether they are monetary or symbolic. Someone has something of value that can be traded for something else.
Religious Values:	These values have to do with piety, purity, and restraint. Mysticism, mystery, fear of the unknown may be included amongst these values. These values tend to be related to salvation, damnation or judgement by a higher deity.
Aesthetic Values:	Any value related to the appreciation of beauty. If something is seen as elegant, simple or desirable (or the opposite) with respect of an emotional reaction, then Aesthetic values are being used.
Military Values:	These values involve the organization towards the defense or attack. This defense/attack is not limited to a geographic area. It can also involve discipline, resilience and pushing through difficulty.
Technical Values:	These values have to do with skill, trades or building. These values require the production of something that has a use.

Modified definitions of the Value Systems by Echeverría [3].

As part of this process, the coders assigned a thematic title to how value systems manifested in the text. Coding was compared and discussed among the coders. A third coder resolved disagreements between the authors regarding the passages' value systems and thematic titles. Once the coders were familiar with the process, they repeated it for all selected articles. Examples of quotes for each value system and their main manifestations are listed in Table 2. Relationships between codes were established, and discussion topics were built accordingly using Atlas.ti version 8.4.4. The most important value system covered 75 % of the quotes.

**Table 2:** Examples of representative quotes of the most common value systems and their manifestations.

Value Systems	Value Manifestation	Example
Basic Values	Agency and Autonomy	“Two major assumptions guide the social cognitive career theory: (a) People have the capacity to exercise some degree of agency, and (b) individuals contend with several factors that strengthen, weaken, or override personal agency” [19]
	Capability approach to justice	“(STEM) graduates to play an integral role in addressing challenges for the human good, including eliminating severe inequities and injustice around the world” [40]
Economic Values	Transactional value of course grades	“Math anxiety is associated with reduced math achievement scores and a variety of negative outcomes including an aversion to math (Ashcraft, 2002). Math anxiety is also related to more negative personal views of math.” [10]
	Perceived value of science	“Task value is conceptualized as multifaceted, with individuals valuing tasks or domains for multiple reasons including the personal importance of a task or domain because of its relevance to their personal and collective (or social) identities (i.e., attainment value). Attainment value in particular is conceptualized as a central, defining component of an individual's personal and collective identities.” [12]
	Capability approach to justice	“Not many will dispute the enormous impact scientific and technological development has had on parameters of the human condition, including increased standards of living, life expectancy, health care, among many others.” [40]
Epistemic Values	Science practices in the teaching-learning process	“In sharing their ideas for an experiment with peers or instructors they have an opportunity to demonstrate their competency with science practices and be recognized for scientific work. This recognition, in turn, may help to strengthen students' identification with the scientific discipline.” [34]
	Identifying as a scientist	“Undergraduate students who begin a semester feeling unsure about their science abilities may be especially vulnerable to instability in their science identities.” [12]
Political Values	Capability Approach to Justice	National priorities in the U.S. have also focused on addressing the disparities in STEM degree completion rates among different groups. Though interest in pursuing STEM degrees has steadily increased in the last decade across all ethnic groups, persistence to degree is low and some groups persist at disproportionately lower rates.” [34]
	Political Involvement of Scientists	“Latina students who were more academically involved on campus had greater STEM career self-efficacy.” [19]
Social Values	Recognition and Success	“An individual's expectancy for success and perceptions of value are key proximal predictors of achievement and choice behavior” [12]
	Identifying as a scientist	“Contemporary expectancy-value theory (Wigfield, Tonks, & Klauda, 2016) highlights the key role of identity-related motivation processes in predicting students' achievement and choices (Eccles, 2009).” [12]
	Racism and Social disparities	“Under-represented minority students were more likely than racial/ethnic majority students to begin college with somewhat lower science identity.” [12]
	Social influences	“A key turning point in my relationship to math was when I got a tutor. This was important because it helped my math skills dramatically. My tutor was very knowledgeable and explained everything to me step by step. My grade in my math class got a lot better after getting a tutor.” [10]

## 3 Results and discussion

The analysis has three components: I) a quality assessment of state-of-the-art STEM education, II) an ethical meta-analysis and the axiological landscape of STEM programs, and III) innovation by translating knowledge through good teaching practices in STEM education.

### 3.1 Quality assessment of state-of-the-art STEM education

#### 3.1.1 Search strategy results

Fig. 1 summarizes the methodology used in this study. The search yielded 595 articles. Fewer than 30 % of the articles were obtained from the Web of Science [23], nearly 65 % from Scopus [24], and 7.5 % from PubMed [25]. There were 109 duplicates, and only 131 hits were relevant to the research question (Fig. 3). Most of the retrieved articles were from Scopus [24], whereas Web of Science [23] and PubMed [25] together accounted for less than 40 % of the retrieved literature. This is likely because of the nature of such databases, in which Scopus condenses a broader number of research topics and authors, publishing in many indexed high-quality journals. PubMed integrates articles that mainly target the biomedical sciences. The Web of Science offers a collection of articles published in high-impact, high-quality journals, explaining why nearly one-third of the articles were from this database.

**Fig. 3:** PRISMA Flowchart that depicts the steps followed in the systematic review process including reasons for article selection.

#### 3.1.2 Screening results

After reading the titles, 73 articles were found to be relevant to the research questions. Only 23 articles met the inclusion criteria after reading the abstracts, materials, and methods. Table 3 summarizes the details of each study. The most common reasons for excluding articles were not having an undergraduate degree (38 %), not being an observational quantitative or mixed-method study, or being a qualitative study (26 %). More than 5 % of the articles were excluded for not exclusively studying STEM undergraduate tracks or for not having measures, attitudes, or values as outcomes (Fig. 3). Most of the selected articles (87 %) were cross-sectional quantitative studies, two were qualitative studies, and one was a mixed-method study.

**Table 3:** Summary of selected articles.

Article	Research Question	Design	Target population and sample	Research Instruments	Timing of Application of Instruments	Main Findings	Strengths	Limitations
Black & Hernandez-Martinez, (2016) [17]	How does science capital and mathematics of students mediate between student background and career choice?	Case Study	2 cases chosen from 50 participants in a larger story. One student was female from a middleclass family, and another student was a male from a privileged background. Both were majoring in Physics.	Questionnaire to explore reasons for choosing career, aspirations for future, experience in university, and perceived effect of ethnicity, gender, SES on academic trajectory. Narrative analysis of interviews focusing on science capital, cultural capital and identity.	Beginning of Year 1 End of Year 1 During Year 2	- One of the two students liked doing science and was immersed in it from a young age; the other participant was just studying science to get a good job in finance. - Both participants reported the importance of maths in their program.	- The choice of cases in the study is in line with the research question. - Instruments and questions are pertinent. Findings are consistent with literature	- Validation of questionnaires is not very clear. - Possible instability of narratives according depending on many factors.
Castellanos, (2018) [19]	What psychosociocultural factors affect Latina's career decision-making process in STEM?	Cross Sectional	460 female Latinas in their second year of college or higher. Attending a predominantly white selective institution in California. Family income between $40,000.00 to $70,000.00. Mostly first-generation students.	- *Marianismo* (Self-sacrifice) Scale - Latina Strength Scales - Pre-college Maths and Science Performance - SAT Maths scores - STEM Career Self-efficacy and Interest Scales (Adapted from Byatz) - Perception of Barriers (Adepted from McWhitler) - Major choice goal scale	Not clear	− 13 latent constructs from 60 variables. - SES and generational status are positively correlated to maths and science learning experiences (MSLE). - MSLE also positively correlated with having STEM self-efficacy (SSE). - SSE is correlated with academic involvement, interest and having STEM career goals (SCG). - Faculty plays a role in increasing interest. - Undesirable classroom climates may be an obstacle for developing interest and SCG.	- Use of a variety of constructs and questionnaires. - Large sample size - Validation of questionnaires. - Findings are consistent with literature.	- Possible attrition bias due to the large number of questions. - Participants receive an award for participating and it is not discussed whether this may bias results.
Garibay, (2018) [40]	What makes STEM students get involved in social and democratic projects after college?	Longitudinal	6341 participants, 47 % female. Above a third of the students had a parent working in STEM. 10 % black, 10 % Latina/o, 3 % American/Alaska native, 14 % Asian/Pacific, 61 % white, 2 % other	Survey: − 2004 social agency − 2011 social agency - Faculty Civic-minded values - Faculty Student-centred pedagogy	Applied to faculty and students 7 years apart. Unclear at which point of the semester.	− 17.5 % had social agency (SA), 36 % felt that conducting meaningful research (CMR) was important, 27.6 % that CMR is not important, 64 % that CMR is not/marginally important. - Women of underrepresented minorities (URMs) had significantly more SA and valued CMR than white counterparts. - Freshman SA and CMR predicted 7 yrs later. - Engineering students scored low in SA and CMR. - Participating in undergraduate research is associated with higher SA and CMR. - Socioeconomic Status (SES) negatively correlated with valuing CMR. - Health professionals and people in a STEM position tend to value CMR but have low SA. - Schools may be promoting CMR, but not political involvement	- A large number of variables are analyzed.	- Data limited to what was available in the surveys. - Impossible to elaborate on reasons why these trends were obtained
Hilts, Part, & Bernacki, (2018) [18]	How do URM's relatedness and competence influence completing a STEM degree? How does social support affect belonging in STEM programs?	Longitudinal	406 invited students taking an anatomy course, 206 participated. 73.3 % female, 24.8 % first generation students. 34.5 % URMs.	- Perception of competence scale - Relatedness scale (adapted from Robnett). - Friends’ and peers' value of STEM scale. - Contact with STEM peers (vicarious experiences). - Intent to leave STEM program - Previous anatomy knowledge test (pre-test).	On the 1st, 8th, and 15th weeks of a 15-week course.	- Small correlation between pre-test and feelings of competence. - Males and females, URM and non-URM, first generation and non-first-generation students showed similar STEM learning competence. - Contact with peers in STEM associated with STEM relatedness - STEM relatedness was negatively associated with final grade. - Contact with classmates (in-person) associated with feeling competent. - Intent to leave negatively correlated with competence	- Large number of participants.	- Participation weighed on final performance. No discussion of how this affects the results. - A large number of constructs measured may bring attrition. - Does not mention reasons why students didn't follow up
John, Nelson, Klenczar, & Robnett (2020) [10]	What are the life-story math narratives of undergraduate students? How do these narratives vary depending on ethnicity and gender? How are the narratives and career selection associated?	Mixed methods	343 students from a southwestern university taking an introductory psychology course. Ages 18–24. 66 % women, 33 % men, 0.5 % transgender men, 0.5 % undisclosed, 36 % white, 27 % Hispanic/latinx, 21 % Asian/Pacific Islander, 11 % African American, 2 % mixed race, 1 % Native American, 1 % other, and 0.5 % Middle Eastern	Math-specific version of McAdams' life turning points. Math Anxiety scale (Hopko) Math-self expectancy (Watt, 2012) Math value (Watt, 2012) Future math plans (open-ended)	Not clear	- Over half of the participants gave good turning point narratives. - Nearly 30 % of the participants provided with redemptive stories about maths. - Contamination, consistently positive, and consistently negative narratives appeared in 15 % of the cases each. - Turning point stories showed that students experienced issues with maths differently: a low mark may motivate some students or discourage others. - Course instructors may be catalyzers of redemptive or contamination stories. - Consistently negative narratives were associated with avoiding activities that require maths in the future. This was a less common effect in students with other narratives	- Mixed methods approach. - Correlates stories and life story turning points with academic outcomes	- Unclear moment of interviews and instrument application.
Perez et al. (2019) [15]	How do competence beliefs, task value, and perceived costs explain motivational profiles in STEM students? How do motivational profiles explain short and long term STEM academic achievement and course completion? How do these results vary between URMs and genders?	Longitudinal	A subsample of a cohort of 1st year students taking a chemistry course in a trial. Subsample of 600 students did not receive intervention. 50.5 % female, 30.6 % Asian, 48.0 % White, 7.6 % African American, 7.1 % Latino, 6.2 % multiracial. 4 % first generation students	Science competence beliefs Science Task value Science perceived costs	7 weeks into semester, grades at the end.	− 3 profile model had the lowest Bayesian Information Criterion (BIC). - Competence beliefs score was positively correlated with task value scores. - Perceived effort cost was negatively correlated with task value scores - Opportunity cost and effort costs were positively correlated. - Higher competence was associated with lower cost. - Three profiles: (A) Moderate self-expectancy, task value and perceived costs; (B) Very high competence and task value, low effort cost; (C) High competence and value, moderate-low effort cost.	- Use of Latent Profile Analysis permits to do a person-centred analysis, rather than a variable centred one. - Findings are consistent with literature.	- Participants were given a monetary reward, which may bias the results. This is not further discussed.
Robinson, Perez, Carmel, & Linnenbrink-Garcia, (2019) [13]	How does belonging different identity patterns predict performance in a 1-semester chemistry course e and STEM status?	Longitudinal	1669 undergraduate students enrolled in a chemistry class. 55 % female, 13.7 % first generation students, 73 % White, 13.7 % Asian/Asian American, 6.0 % Black, 1.9 % Hispanic or Latinx, and 5.9 % multiracial, Native American, Pacific Islander or other.	- Science Identity Questionnaire (Robinson, Peres, 2018) in T1, T2, and T3. - Science Academic Perceived Competence (T2) - Chemistry exam score (T3)	During the (T1) 2nd, (T2) 8th and (T3) 14th weeks of a 15 week course	- Repeated measures of science identity were correlated between each other, and with perceived competence and final exam score. − 60 % of the students remained in a STEM program after one semester, 29 % remained in a non-STEM program; 4.4 % switched between a STEM to a non-STEM program, and 5.8 % switched from a non-STEM to a STEM program. − 3 Science Identity categories: (A) Starts with high Science ID and remains more less high, (B) Starts moderate Science ID and moderately increases over time and (C) Start with moderate initial Science ID and declines slowly over time. - Most students (53.8 %) were in class (A) - URMs were more likely than white or Asian to be in (B) than (A) but as likely to be in (C). - First-year students were more likely to be in (A) than in (C) when compared to upper class. - Higher competence beliefs associated with belonging to class (A). Students in class (A) were more likely to get a higher final exam grade and to remain in STEM.	- Robust person-centred analysis. - Large sample size.	- Participation was awarded with course credit. This could bias results and is not discussed. - In this school, STEM was only pure sciences and engineering; life sciences were not considered STEM
Robinson, Perez, Nuttall, Roseth, & Linnenbrink-Garcia, (2018) [12]	How does belonging different identity patterns predict performance in a full STEM program?	Longitudinal	1023 students in a STEM program, 58 % female, 25 % white, 43 % Asian, 13 % African American, 11 % Hispanic/Latino, 8 % multi-racial or other.	- Science ID: Self-Report scale designed by Pugh et al. and Attainment Value Scale (Conley) - Competence beliefs: two questionnaires by Estrada and Midgley. - Science involvement after graduation: Self-report question.	Yearly during 5 years	- At all time points, Science ID, Self-efficacy, and Perceived competence were positively correlated. - Model with 3 categories (lowest BIC) of Science Identity found in students: (A) Quadratic model with negative second-degree coefficient. Science ID grows fast at the beginning but slows down (B) Relatively low science ID at the beginning, remains stable through time, and (C) is a quadratic model with a rapidly decreasing science ID (second degree coefficient is positive). - Model intercepts are statistically different (A) > (B) > (C). - Women are twice as likely as men to be in (B) than in (A). - URMs are two times more likely to be in (C) than in (A) when compared to the majority.	- Robust person-centred analysis. - Large sample size.	- Loss of follow-up
Rosen & Kelly, (2020) [31]	What are the similarities and differences between undergraduate students' beliefs regarding the epistemological value of laboratory tasks, socialization, and help seeking in the physics laboratory when comparing students taking an in-person laboratory course, and those working in an online laboratory course?	Quasi-expertimental, observational quantitative study	998 undergraduate students enrolled in calculus-based introductory physics studying at a public university (50.5 % male and 49.5 % female) of which 41.3 % classified themselves as Asian, 9.5 % as Black/African American, and 13.1 % as Hispanic/Latino	Questions were taken from the E-CLASS survey and the Laboratory Classroom Environment Instrument for Senior High School Science. Additional questions were designed to collect data on affective constructs. After administration of a revised survey to the main sample, additional items were removed to maximize validity and construct reliability. (24 questions in the final survey)	During the second half of the semester	- Online and in-person students demonstrated statistically similar perceptions of epistemological beliefs about laboratory work. - In-person students expressed higher positive perceptions of the value of socialization compared to online students. - In-person and online students did not indicate significantly different perceptions of seeking assistance. - Men showed higher composites on their epistemological beliefs than women. - No significant differences between men and women about socialization - Women reported greater willingness to seek assistance than men - Men and women didn't report different views of epistemology, socialization, and help seeking depending on the type of course in which enrolled.	- Findings are consistent with literature. - Survey used had adequate overall reliability - Sample size for factor analysis met the excellent-level criterion for a three-factor solution	- Data collected from a single research university - Correlation between self-reported beliefs and physics performance was not measured - Randomized controlled study would allow the exploration of outcomes with minimized selection bias
Sax, Lehman, Barthelemy, & Lim (2016) [32]	How has incoming college women's intent to major in physics changed over the past four decades? How have the career aspirations of women who plan to major in physics changed over the past four decades? What individual characteristics correlate with women's decision to major in physics vs all other fields?	Mixed methods	- 1st analysis: 4 577 098 female first year-college students - 2nd analysis: 4 375 369 female first year-college students - Regression analysis: (1) 399 766 female students from across all majors and (2) 65 993 female students who planned to major in any of the STEAM fields	CIRP Freshman Survey (1971–2013)	Each year from 1971 to 2013	- Women´s interest in majoring in physics remains low and is lower than their interest in other STEM majors. - Research scientist is the most popular career choice among female physics majors - The number of female physics majors undecided about their career plans has increased over time - Female physics students present a distinctive profile as compared to women from all other majors and in other STEM fields - Women who intend to major in physics are more confident about their math abilities, desire to make theoretical contributions to science, attend college for educational reasons and aspire to either master's Ph.D. degrees.	- Large sample size - Large collection of variables - Long-time perspective	- Unable to address whether or not that intention actually leads to completion a physics degree - Do not capture any predictors of majoring in physics that may be unique to community college students
Simon & Nene (2018) [41]	How are masculinity/femininity and classroom climate related to choosing STEM majors in women?	Cross-sectional	752 students 19 years or older in a public university completed the survey. A subset of 425 majoring in a STEAM field. 45 % female, of which 52 % were in Physics, Maths or Engineering (PEM). Males outnumber females in PEM 2-to-1. -Nearly 72 % of STEM majors were in PEM	- Academic Climate - Bem Sex Role Inventory (BSRI) Masculinity-Femininity - Occupational values	Not clear	- Males in PEM had significantly lower femininity than females in PEM. - All individuals in life sciences exhibit higher altruistic/communitarian values than students in PEM. - Females in PEM report being treated unfairly more often than males in life sciences. - PEM students presented more conservative gender attitudes than the other students - Gendered personalities seem to have no effect on STEM choice. - Females in life sciences tend to feel a more welcoming environment than females in PEM. - Males with high masculinity perceive a welcoming climate in life sciences, while females with high masculinity do not.	- Analyzes the topic of gender in STEM from a more sophisticated point of few than just sex.	Unclear sample description and time of application of the
Starr et al. (2020) [34]	What is the effect of different science classroom practices in STEM motivation and career aspirations	Longitudinal	1079 students taking a different biology course. Some enrolled in small active learning sections and some in large lectures. Around 38 % were Asian, 30 % White, 25 % Latino, 3.7 % African America.	- Frequency of science practices (Buck) - Recognition as a Scientist - Classroom Climate (Stake and Mares and Leoper) - STEM motivation (Kosovich) - STEM career aspirations. - Non-STEM motivation (Same as STEM motivation but substituting STEM with non-STEM)	First two weeks (T1) and last two weeks (T2) of a 10-week semester.	- URMs had a lower GPA and biology course grade than the majority. - Classroom climate was associated with increased motivational variables in T1. - Performing Research Practices (RP) was associated with higher scientific recognition and better classroom climate, but not with STEM career aspirations. - Recognition as a scientist mediates the relationship between performing RPs and changes in STEM ID - Classroom climate mediates the association between recognition as a scientist and changes in STEM motivation.	- Large number of variables were analyzed	- Possibility of attrition bias is not acknowledged or discussed.

#### 3.1.3 Quality assessment of articles following the PRISMA approach

Thirteen articles were excluded for using quality assessment instruments. Two articles were added manually because of their relevance to the research question and approach to justice content [31,32]. The average score for the 23 articles was 65 %, with a coefficient of variation of 30.5 %. The quality score of the selected articles was 77 %, with a coefficient of variation of 11 %. The characteristics of the selected articles are summarized in Table 3.

A wide range of publications address the issue of values and attitudes toward STEM teaching at many levels; however, the present review focuses on analyzing and discussing baseline value systems without any intervention. While the authors recognize that values and attitudes stem from early life and that the most effective intervention for shaping an innovative STEM society should occur from family upbringing and early schooling [33], it is crucial to address and correct the voids in STEM-related values among undergraduate students as much as possible. Therefore, several articles on early STEM education were excluded even if they met the inclusion and exclusion criteria. Moreover, although many articles offered insightful and vital information on STEM attitudes and values, strict standards were applied to ensure that the studies were homogeneous and relevant to the research question. Table 3 summarizes the articles included in this review.

### 3.2 Ethical meta-analysis and the axiological landscape of STEM programs: do STEM education values foster innovation?

An ethical meta-analysis is a novel qualitative or mixed-method methodology that complements any systematic review by adding an in-depth axiological, behavioral, attitudinal, or virtue evaluation of the literature. While a typical meta-analysis reviews the quantitative results of several articles in a systematic review to obtain a pooled estimate, an ethical meta-analysis qualitatively explores the narrative of all the articles. It evaluates the value systems that emerge in all literature to build an axiological landscape and helps identify gaps that could be solved through cross-functional value-based approaches. The ethical meta-analysis results from a hermeneutic study of the narrative of the selected papers.

The results of the ethical meta-analysis can be grouped into three subtopics on STEM education: 1) ethical perspectives, 2) emerging values and axiological frameworks, and 3) ethical dilemmas. The subtopic regarding ethical perspectives shows a straightforward consequentialist/utilitarian approach to STEM education. The second subtopic of the axiological framework shows that values must be more explicit in the literature and that innovation as a goal of STEM education is addressed only as a tangential issue.

None of the value systems proposed by Echeverría were excluded from the analysis, but only four were the most relevant. Basic, economic, epistemic, political, social, and technical values were the most prevalent (central) value systems in the STEM literature. The remaining value systems appear to be secondary. Juridical values appeared in only one of the analyzed articles and were irrelevant to any discussion in the paper. Fig. 4 shows the value systems in decreasing order of coding frequency. This figure shows that nearly 75 % of the coded value systems can be attributed to four systems, social, economic, aesthetic, and epistemic, of which social values appeared to be the most central in the articles analyzed. Finally, the literature addresses an implicit ethical dilemma in STEM education: student evaluation in an unequal context. A thorough discussion of each subtopic was developed.

**Fig. 4:** Absolute and accumulated frequencies of coding of each value system in selected articles.

#### 3.2.1 Innovating STEM education by applying maximal ethics

There are three fundamental approaches to ethical discussions: 1) deontology, 2) aretology, and 3) consequentialism. Deontology establishes the codes of conduct that serve as a moral compass. In this approach, the code of conduct determines a duty for each person, and moral goodness implies fulfilling these duties regardless of the consequences. Aretology or virtue ethics is based on the concept of “phronesis,” which implies that each philosophical object can be put in its right place. Virtue ethics emphasize bringing value to life and placing it in the right place (virtuous behavior). Therefore, people who behave virtuously always gravitate toward moral goods. Finally, consequentialism or utilitarianism assigns moral goods to actions depending on their consequences. This implies conceptualizing and anticipating most of an action's possible consequences and establishing the best course of action that benefits the most people (or harms fewer people) [33].

Although the literature shows deontological and aretological directions, the consequentialist approach is the most favored because of its intuitiveness. To avoid depersonalization, STEM education is viewed as a moral good because of its concrete repercussions in daily life. Discussions on the usefulness of STEM disciplines and STEM education content highlight the economic value system of Echeverría. It has been consistently mentioned that students perform better in STEM courses when they see value in their studies and a direct connection with their personal lives. As mentioned earlier, one of the many things a student may value in a course is its relevance and applicability [10,12,13,15,34,35]. The value science was given importance in seven articles [10,12,13,15,17,18,31]. One exciting aspect highlighted in the literature was economic value, which is the “perceived value” and “perceived costs” of studying in STEM tracks. Perez et al. [15] described the perceived value of science as follows:

“In terms of task values, three different kinds of positive task values are included in the expectancy‐value model: (a) interest value, the anticipated enjoyment of a task or interest in a domain; (b) attainment value, the perceived importance of a task to one’s identity; and (c) utility value, the subjective value of a task for attaining an extrinsic goal such as a career goal.”

Conversely, Perez et al. [15] described the perceived costs of STEM as follows:

“[…] (a) effort cost, perceptions of whether the time and effort needed to be successful on a task is worthwhile; (b) opportunity cost, perceptions of lost opportunities to engage in other valued activities; and (c) psychological costs, perceptions related to fear of failure and anxiety associated with engaging in the task.”

STEM's perceived values and costs are tied to another fundamental manifestation of economic value: providing necessary job skills. Students' preferences for specific topics and their tolerance of difficulty can partly be attributed to their future usefulness. The following excerpt from an interview by Black and Hernandez-Martinez [17] depicts a utilitarian approach toward learning STEM from a physics student:

“Particularly, Elton’s awareness that a Physics degree has exchange value in terms of getting a good job indicates his awareness of this system of exchange (symbolic capital). He believes that studying Physics will ‘prove he is clever’ and that he is ‘able to solve real life problems.’ despite this, he states that in the end his future will not be in Physics: ‘You do what pays’.”

Designing STEM course content is a cumbersome task because it is not always evident which topics are pertinent to attaining the goals of STEM education [36]. Because STEM education goals are manifold, considering it from an integral standpoint allows expanding its scope, aims, and evolution by fostering the development of an axiological technoscientific culture instead of just teaching the content needed for a job. This approach humanizes STEM practices.

Moreover, all individuals have reasons to study and should have the agency to choose whatever will help them fulfill their lives. Students whose ambitions are not academic may justifiably question the relevance of university or secondary education curricula. Therefore, several countries have multiple-track secondary education systems, where students pursue either academic or vocational education early in life [37]. Thorough nonbinding evaluations assist in this choice, and students may change tracks later in their careers [38]. When the ends of the educational system match those of the students, there might be less resistance and effort to acquire the value of the discipline. However, these systems exhibit several limitations. They can be criticized for cultivating elitist societies [36] when applied to countries with high inequality. This is in line with Nussbaum's idea of cultivating justice with a capability approach, where every person is truly able to pursue his or her own ends without structural obstacles.

Usefulness and relevance are related to personal preferences, career ambitions, and transient disciplinary trends. A nutrition and dietetics student looking forward to obtaining a job in the food service sector may question the relevance of studying metabolic pathways in depth but may place high value on food science courses. Conversely, immunonutrition is currently perceived as a more relevant topic due to the SARS-CoV-2 pandemic in 2020. Even those students who attend schools of applied sciences or trade must take challenging STEM courses that may not seem relevant at first but will be an important foundation for later courses. This is even the case in medical schools, where the relevance of the basic sciences is continuously challenged [39].

Our proposal for STEM education is based on the principle of maximal ethics. This approach is called integral ethics. In this approach, we consider all the values of the three main ethical theories mentioned above, and the core vector redirects the values to give sense and a hierarchical meaning. For example, we care for people and their ends (aretological) in STEM education. However, we believe that the student knows and respects scientific-technological normativity (deontological), and, finally, we desire cost-effective outcomes (utilitarian). From this integral perspective, the dimensions of STEM education include cultivating students with creativity, the ability to grasp the future, and taking risks to favor innovation and social responsibility.

#### 3.2.2 Emerging values, axiological horizons, and innovative frameworks of STEM education

A summary of the axiological landscape of the STEM literature is shown in Fig. 5. Social values appear at the center and are supported by basic, economic, epistemic, and political values. All other value systems appeared in the literature but were not central to the discussion of STEM education. Table 3 complements Fig. 5 by showing the most critical ways each system appears and a few examples of how this manifests within a particular value system. The capability approach links social, economic, political, and basic values. The social aspect of the capability approach to justice is entrenched in the discussion of inclusive and accessible STEM education and student recognition and success. Social and epistemic values are linked by scientific identity, which can be discussed from a capability perspective.

**Fig. 5:** The axiological landscape of literature in STEM education. Social values appear as the central item in the analysis, but they do not appear alone, they are interconnected in cascade with other value systems.

Several contextual variables (such as social influences, gender roles, teaching styles, and regulatory frameworks) may modulate how well an educational system promotes comprehensive STEM education. The following subheadings (3.2.2.1 to 3.2.2.4) show a full description of how these value systems are related and how they agree with other studies.

##### 3.2.2.1 Social values are at the center of the axiological discussion in STEM education and are linked to other value systems through the capability approach to justice

The most cited manifestation of value systems in the literature is the capability approach to justice, which aims to distribute goods equally according to the needs of each person and seeks to pave the way so that everyone is able to achieve their own wellbeing and life goals [40]. This manifestation appears to be tied to three value systems: basic, economic, and political. The capability approach to justice was the most common manifestation of basic values in 9 of the 12 articles [10,13,14,17,19,31,32,34,41,42]. The capability approach to justice was also the most common economic value manifestation in eight papers [13,14,18,19,31,32,34,41] and the political value manifestation in all articles. The following quote exemplifies how the capability approach to justice is related mainly to political values while underscoring basic social and economic values [34]:

“National priorities in the U.S. have also focused on addressing the disparities in STEM degree completion rates among different groups. Though interest in pursuing STEM degrees has steadily increased in the last decade across all ethnic groups, persistence to the degree is low, and some groups persist at disproportionately lower rates.”

Starr et al. [34] emphasize political values as essential for addressing disparities in STEM education, which is important for the economy and society and reflects the importance of human dignity (basic values). This quote implies that some sectors of the American population cannot pursue STEM degrees for the multiple reasons that drive educational policies. One quote from Simon and Nene [42] describes how women struggle to be included in STEM. The authors attributed this to the cold atmosphere in STEM that curtails women's opportunities and prevents them from accomplishing their goals. This quote underscores basic and moral values [42]:

“Although women have advanced considerably in science achievement, course taking, degrees earned, and professional positions held over the past four decades, most of this growth in female representation within the sciences has been confined to the life sciences while women’s representation in physical, engineering, and mathematical (PEM) sciences remains recalcitrantly low.”

The capability approach to justice is valuable for analyzing development and welfare issues and political and philosophical questions related to social justice and well-being. This theory allows us to conceptualize inequities and differences in development between groups [43]. This approach provides the basis for analyzing and developing goals and objectives in the STEM education context [40,43].

According to this framework, focusing on people's agency and autonomy is the key to achieving a successful society. This fact is continuously underscored in the literature, where feminine traits and minority status appear to block development in STEM disciplines [[13], [14], [15],^17^,^19^,^42^]. Simon and Nene [42] state that women in STEM tend to gravitate toward biomedical domains, where a type of maternal altruism is exercised, as opposed to physics, engineering, and mathematics.

Nussbaum [40] argued that women's career choices may be heavily influenced by an unfair context that prevents them from exercising full agency. Simon and Nene [42] describe a ‘chilled climate’ in the scientific domain that is not inviting for women. Moreover, Castellanos [19] added that women with Latin American backgrounds from more traditional families are often ready to sacrifice their scientific careers to care for their families.

“Latina students with higher socioeconomic status, faculty support, and academic involvement were more likely to have STEM career goals. Those who perceived their classroom climates as hostile and had higher self-sacrifice values were less likely to pursue STEM career goals.”

The following quote from Castellanos [19] describes how undergraduate students may weave religious, social, and economic values when choosing a course of study:

“Close familial relationships often served as a major source of support and encouragement; Latinas also reported difficulties balancing familial pressures and career goals […]. For example, Latinas described feelings of guilt associated with leaving home to attend college and not contributing to the family finances, as well as pressure to be a positive role model for younger family members […].”

Latinas in the US may face a dilemma in which they must weigh religious and social values against epistemic and technical values [19]. Any decision is satisfactory if it is completely free and is not influenced by any sociocultural or economic constraints (including the need to work from an early age).

Military values, which nurture a vertical and hierarchical culture, also underscore these inequities. Many disparities in access to STEM may be related to the replication of masculine roles and military authority. Historically, men have tended to choose careers that involve power, whereas women have been more involved in nurturing and caregiving professions [44]. These preferences may be culturally and socially shaped and have been identified early in education. The following quote by Sax et al. [32] shows how gender differences are introduced during K-12 education, creating a gap in STEM capital for women:

“Students' K-12 experiences have been shown to impact their decision to pursue a STEM field in college. Differences in men’s and women’s academic preparation for STEM coursework in college stems from differences in their K-12 experiences. For instance, as discussed earlier, women tend to take fewer advanced math and physics courses in high school, which leaves them less prepared than men to pursue STEM majors in college.”

Military values appeared in only five articles, with multiple manifestations. The most common manifestation in the three articles was the replication of masculine roles in STEM [13,32,42]. The two remaining articles emphasized the role of authorities or authority groups in learning STEM [10,41]. Historically, war and masculinity have been linked. There has been much debate on how and why these two constructs are related; however, it has been hypothesized that masculinity provides the foundations that allow war to be explained and justified as a cultural practice [45]. Therefore, it is not surprising that many STEM fields replicate masculine structures that may not appear in people with feminine traits [42].

In contrast to military values, religious values underscore the more humane traits of STEM. Two studies showed that commitment, patience, selflessness, altruism, service, and care for living things were important manifestations [19,42]. According to five articles, the most common manifestation of religious values was students’ ability to achieve the greatest good [10,18,31,32,41]. Religious values shape the idea that the end of technoscience is the good of humanity and the planet.

Nussbaum [40] emphasized the concept of agency as the primary goal of the capability approach. Agency and autonomy are polyvalent manifestations of basic, economic, epistemic, social, and technical values. Agency and autonomy appear in the literature in many different contexts and are mentioned 58 times. In more than 22 % of the cases, this code was associated with the capability approach to justice. Perez et al. [15] described a context in which underrepresented minority (URM) students struggle to complete STEM programs:

“URM students were most likely to be classified into the Moderate All profile and were least likely classified into the Very High Competence/Value-Low Effort Cost profile, suggesting that URM students may be more likely to develop a profile of science motivation beliefs that is less conducive to persisting in STEM, perhaps as a result of systemic barriers faced by URM students in their early college experiences […].”

URM students may have different agency to pursue a STEM degree than other more privileged students. This restricted capability contradicts human dignity and basic values. A student who is in*capable* of pursuing a STEM career will not acquire or improve her scientific knowledge, suggesting a relationship between a capability approach to justice and epistemic values. Since technological values materialize as epistemic values, an unfair distribution of capabilities compromises this value system. Starr et al. [34] argued that research experience can motivate students who feel they need more capabilities to pursue a STEM degree.

“Providing research experiences to students is widely regarded as a means of advancing more students from underrepresented groups into STEM, and studies have demonstrated success. Some studies have established more concretely that the positive outcomes of research experiences arise from students performing science practices, which led to science self-efficacy, identity, and motivation to pursue a STEM career […]. In addition, laboratory courses that are more reflective of authentic science seem to be particularly beneficial for retaining women […] and underrepresented racial-ethnic groups.”

A capability approach to justice is also associated with aesthetic values because recognition, success, and agency go hand in hand. Recognition and success were coded 70 % of the time, while agency and autonomy were also coded. Hilts et al. [18] stated that academic achievement in STEM courses is often associated with perceived capability.

“Positive perceptions and beliefs about learning and the availability of social support are known to predict key learning outcomes including engagement and achievement.”

Help, guidance, and peer support have been considered helpful in overcoming epistemic shortcomings in different settings. However, Hilts et al. [18] question its effectiveness in underrepresented and vulnerable students:

“Academic support such as training students' learning skills, providing tutoring on course topics, and academic writing support can benefit the achievement of all students, but less is known about the underrepresented student experience and the kinds of additional supports they may require.”

Helping and supporting vulnerable people may be considered religious. This is how religious values are related to the capability approach to justice and may foster STEM.

Exposure to STEM varies across families and cultures. Black and Hernandez-Martinez [17] described this exposure as a privilege that can be considered a form of capital. STEM capital can be defined as qualifications, operative knowledge and understanding, social contact, and access to STEM disciplines [17]. STEM capital theory goes hand in hand with the capability approach to justice, with some students being more capable of decisively pursuing their scientific goals than others because of greater exposure to science in life. This is problematic because people who have accumulated more STEM capital will be able to produce and accumulate even more, and will be more capable of having access to other forms of capital. The following quote illustrates that students may even display different motivations for accumulating scientific capital [17].

“We conclude that there is a need to reconceptualize science capital so that the dialectic relationship between its exchange and use value is theorized more fully. Whilst some students may access science capital as a means to accumulate capital (e.g., qualifications) for its own sake (exchange value), others appear to recognize the ‘use value’ of science learning and knowledge and this produces different forms of engagement with science (and mathematics).”

Finally, the issue of social inequities generating unfair capability distribution must be considered, especially because the lack of access to technology further disempowers vulnerable populations, as expressed by Garibay [41].

“Two common explanations for the limited impact of [science and technology] on social equity are that their benefits have been uneven and exclusive […] and that science and technology have often been used in socially and environmentally regressive ways.”

##### 3.2.2.2 Social values are also discussed from the perspective of social influences, social recognition, and success, which are important mediators of attitudes toward STEM courses

Social influence appeared as a node in the networks linking nine value system pairs: aesthetic to basic, aesthetic to religious, epistemic to religious, epistemic to social, military to economic, military to epistemic, military to political, political to epistemic, political to social, and religious to social. The literature emphasizes how social influences and authorities drive students to view STEM as a social and political good, which may also lead students to perceive it as beautiful, appealing or valuable.

The beauty of recognition and success is a vital value system that has emerged in the literature and is classified as a manifestation of social and aesthetic values. Quotes could address the social and aesthetic aspects of success, the lack of success or the social and aesthetic impact of recognition and prestige. The beauty of recognition and success, or the lack thereof, was the most common manifestation of aesthetic value in 10 of the papers analyzed [10,14,15,[17], [18], [19],^31^,^34^,^41^]. John et al. [10] described how negative social experiences produce a dislike of mathematics.

“Contamination stories typically involve experiences of failure, betrayal, and accidents. For example, a student whose enthusiasm for math deteriorates after a negative experience with a math teacher is exhibiting a contamination story.”

The role of social influences has been underscored in previous systematic reviews. According to a systematic review of student attitudes toward STEM, social influences can potentially boost deep approaches to learning and even shift unproductive student identities [35]. The results of this review support this by emphasizing that the interaction of peers, teachers, and institutions can modify technoscientific values in students, even in the later stages of education.

Performing scientific practices in class is one way to foster cooperation, commitment, discipline, responsibility, and the foundations of a technoscientific culture among students. Scientific practices detonate creativity and self-confidence and establish an organizational culture encouraging scientific discussions among peers and instructors. All this must take place in a safe environment where errors are tolerated and innovation is valued. When performed correctly, in-class scientific practices may increase students’ STEM identity [34]:

“When students use science practices in classrooms, they are much closer to feeling that they know what it means to do science. In sharing their ideas for an experiment with peers or instructors, they have an opportunity to demonstrate their competency with science practices and be recognized for scientific work. This recognition, in turn, may help to strengthen students' identification with the scientific discipline.”

One quote by Rosen and Kelly [31] describes how building knowledge in a physics lab results from positive experiences and success, widely mediated by social values.

“Students' epistemological beliefs about the construction of knowledge in a physics laboratory class are often based upon their expectations, classroom experiences, and their measures of success. Communication with fellow students and instructors may contribute to their beliefs about physics learning. In an in-person laboratory course, socialization and help-seeking strategies undertaken by students are often facilitated by students' close, physical proximity to fellow students and teaching assistants.”

Peer support can help students overcome barriers and gain vicarious mastery through experiences [35]. Hilts et al. [18] described this as follows:

“Experiences with equals and more senior peers who serve as mentors also contribute positively to students' experiences of relatedness. Peer mentoring develops from the association of two individuals of equal status with similar qualities.”

While peers are important, teachers, instructors, tutors, and teaching assistants play crucial roles in cultivating, increasing, and even destroying students’ scientific performance and wholeness. In the literature, this appears as maintenance, redemption, or contamination narratives [10]. An example of a contamination narrative by John et al. [10] is as follows:

“A turning point would be in elementary school. We didn't learn a lot of math because our teacher wasn't there and someone else taught us. That person wasn't a good teacher. I think this is why I'm not that good at math and I don't like it.”

Higher education students are not only influenced by their close peers or professors. Students are also immersed in an institutional framework with specific values, attitudes, ends, approaches, and prejudices toward STEM disciplines. Only one article underscored the importance of institutional and departmental influences on students’ technoscientific values. In this publication, the authors argue that students develop social agency and political values (this article calls them democratic attitudes) through socialization within the institution [41]:

“Academic departments can influence a wide range of student outcomes, including students' aspirations, goals, values, and attitudes […] given that students take more courses in the major than in any other field and become exposed to the culture and values of the department through their interactions with both faculty and peers […] there are two critical components that one must consider in order to understand the influence that academic departments exert on their undergraduate students: (1) the specific goals academic departments have for undergraduate education and (2) the means and resources available to achieve those goals.”

However, it is also possible for departments to negatively influence their students, especially when STEM courses are prerequisites for discipline-specific courses offered by different departments. One recurring example is the general and organic chemistry requirements for medical schools in the United States. Students and faculty tend to question the usefulness of such courses, and the medical school curriculum is continuously adjusted to include relevant content [46].

While clinical faculties tend to question the relevance of general and organic chemistry in the medical curriculum, faculty teaching biochemistry-related courses seem to agree that topics such as functional group reactivity, thermochemistry, chemical equilibria, and kinetics are essential principles for medical students [47]. Other authors suggest that the basic sciences, included in STEM, offer foundational knowledge that will not be directly applied in clinical practice but will help “encapsulate” other more complex concepts and build knowledge networks [39]. This debate enriches how STEM disciplines are taught to future professionals. However, no study has examined how this lack of consensus on what should be included in the curriculum affects technoscientific values.

##### 3.2.2.3 Innovation in STEM education: epistemic values are tightly entangled with social values

Epistemic and social values were well connected and form a complex network in qualitative analysis. The two values appear to be close to each other. The most common practice was self-identifying as a scientist [[13], [14], [15],^17^,^19^,^32^], followed by performing STEM-related practices in class (following the scientific method, for example) [10,31,34,42], mastery [10,18], interest in acquiring scientific knowledge [15,32], and the importance of having STEM-literate citizens [41].

Performing STEM-related practices in class is considered a way in which cooperation and collaboration can create vicarious mastery experiences for students and positive social influences that increase technoscientific value. Therefore, they can be viewed as having both social and epistemic value. The retrieved literature addresses other critical social aspects of performing scientific value. The literature mentions that scientific practices include but are not limited to “hypothesizing and explaining results” [34].

When educating future professionals in any STEM discipline, it is crucial to underscore the importance of cooperation, commitment, discipline, responsibility, creativity, and tolerance for errors. This also implies an inquisitive work ethic that values correctness, conciseness, and coherence. These social and epistemic values, along with course quality and course content, have been taken for granted in the literature. A gap in STEM education research concerns how well STEM courses cover specific learning objectives, especially those related to becoming a comprehensive research scientist.

##### 3.2.2.4 Social and political values converge when discussing the social impact of science, lobbying for innovation, and the environmental concerns of science

The literature places little curricular emphasis on how STEM can improve quality of life and how scientists can become involved in democratic and political spheres to influence government guidelines. STEM disciplines are empowering. Currently, powerful societies have knowledge-based economies and can provide solutions to current issues. The gradient in STEM cultures between societies has also deepened the socioeconomic inequities between them [36,42]. Fostering political values among students in STEM disciplines can democratize science and decrease inaccessibility and elitist traits. Moreover, this may motivate others to pursue STEM careers to benefit society and humanity. As discussed, social influences affect students’ technoscientific values and career choices.

Innovation is a means of bringing STEM products to the public. Given the current importance of forming STEM human communities, it is surprising to see little emphasis on technoscientific innovation. Only nine of the quotes in the analysis were related to this topic. Most appeared in Garibay [41], illustrated by the following excellent example:

“Not many will dispute the enormous impact scientific and technological development has had on parameters of the human condition, including increased standards of living, life expectancy, health care, among many others.”

Other quotes were related to educational innovation in STEM courses. An example by Rosen and Kelly shows how technoscientific innovation may improve STEM courses [31].

“The ubiquity of the internet came with innovations in the way science laboratories are conducted. Rather than having to go to a special room with specialized equipment at a specific time, students may conduct entire scientific experiments asynchronously from any location.”

While focusing on education, this quote proposes how innovation may increase the reach of education in remote areas and help democratize STEM disciplines.

Regarding ecological value, Garibay [41] discussed the environmental impact of STEM. This was conducted in the context of scientists performing activities that had a meaningful impact on society and the environment. The only other manifestation of ecological value relates to the context or setting of STEM education [10,18,19,41]. Juridical values are primarily associated with STEM regulations and are only explicit in Garibay [41].

#### 3.2.3 Innovation by discernment of ethical dilemmas in STEM education

In the literature, central values are often paired with equity and social justice. All the actions and decision-making in STEM education that are based on the values systems mentioned above from three ethical perspectives (deontological, aretological and utilitarian) will be referred to as “STEM education ethical issues (SEEI)”. SEEIs in all the analyzed literature emerge primarily because of racial and social disparities. Other critical SEEIs and dilemmas are addressed tangentially, raising an interesting question: To what extent can basic STEM courses be used to discourage students who have not yet developed the necessary competencies and skills [10,13]?

As mentioned earlier, most of the SEEIs that appear in the literature are related to a capability approach to justice; however, Robinson et al. [13] hint at an interesting dilemma in the following paragraph:

“[…] difficult introductory ‘weed out’ courses in STEM fields can present challenges to maintaining high and stable science identities […]. Some students may begin to doubt their ability to succeed or their fit within science when encountering difficult coursework, competitive course climates, or even discrimination and activation of identity-based stereotypes.”

STEM degrees and courses must refrain from replicating oppressive practices that prevent women and URMs from succeeding. Educational sociologists have studied how educational practices and curriculum design may foster education and perpetuate these hegemonic structures. One school of thought believes the current academic environment is designed by those in power, disregarding the fact that it puts minorities, women, and low-income people at a further disadvantage [36].

The fact that higher education highlights disparities in educational quality and capabilities is undeniable. In countries where university/college education is prioritized, students arrive at first-year classes with varying degrees of “university skills.” This variability can be attributed to the privilege and marginalization of students [36], which raises two questions that ignite heated debates in today's educational system: How should teachers proceed when students complete a course without the knowledge and competencies they should have already acquired? What should teachers do for students who arrive on the first day of class without the necessary preparation?

This SEEI benefits from in-depth axiological analysis. Some people believe that the sole idea of evaluation and failure creates a system of classification that perpetuates inequities (Connell, 1992), while others consider that a merit system is necessary. The latter school of thought does not advocate for an unequal and discriminatory educational system but rather a rigorous education that provides content and shapes students’ values and technoscientific organizational cultures early on [48].

If students progress through an educational system without learning content or acquiring competencies, the system loses its purpose. In these systems, inequities in scientific capital and epistemic backgrounds among students have not been resolved. It is unpleasant for students to receive negative feedback or to repeat a course, especially if they cannot develop basic skills due to a disadvantageous background. Nonetheless, removing evaluations and advocating for less rigorous education does not address the root causes of social disparities and further relegates students from disadvantaged epistemic backgrounds while demotivating students who want to be challenged.

Curricula offered worldwide may not be relevant to every person [36]. A system configured with multiple tracks based on the ends of each student can be an excellent solution to this problem if implemented within a state that ensures all opportunities lead to similar outcomes in quality of life.

### 3.3 Innovation by translating knowledge through good teaching practices in STEM education

The literature identifies four stakeholders who play essential roles in developing technoscientific value in higher education: students, teachers, educational institutions, and government institutions. Inequities in access to STEM disciplines are a pending task, particularly because STEM disciplines are not producing results for those who still need to be empowered. Future STEM education should not replicate hegemonic power structures, and higher education institutions should ensure welcoming environments for people from different backgrounds. However, STEM disciplines must encourage a “STEM *ethos*” and an innovation-directed, value-based organizational culture. This remains an important topic to explore in future STEM education research. To achieve this, institutions must emphasize the importance of STEM in reducing inequities and improving the quality of life of all living beings and environments while underscoring a STEM *ethos*. STEM graduates with social agency and political values are greatly needed; however, they are like chairs that are missing a leg if they do not carry themselves in a truly scientific manner.

Based on the issues above, we propose the so-called “virtuous STEM education model.” This model (see Fig. 6) is a value-based innovative proposal. Its main goal is to foster an organizational culture of innovation in students, serve as the cornerstone for educational innovation practices and promote a STEM *ethos* among all stakeholders in STEM education. The model underscores the idea that the four stakeholders are important in developing STEM human capital and distributing responsibilities without burdening any of them. According to the competing values model, each member of an organization (in this case, STEM education) brings their own goals, ends, values, and behaviors, which, as a sum, may or may not foster innovation, depending on which values prevail [22]. Virtue is a quality or trait that supports the development of specific values or groups. Every virtue is a value, yet not every value [33]. The proposed model (Fig. 6) is virtuous because it aims to build and strengthen the virtues that conform to each stakeholder's technoscientific values. This model relies on the idea that values must come to life in the classroom and is based on the values identified in the literature, promoting what was found to be positive and discouraging harmful practices that diminish virtue. The model also appears to foster values that are not emphasized in the literature but are considered necessary for developing technoscientific thought in students.

**Fig. 6:** The higher STEM education culture model. This model focuses on stating and developing goals, ends, values, and behaviors in the four main stakeholders of STEM education: The Student, the Professor, the Educational Institution, and the Government. We propose that following this model could lead to the improvement of techno-scientific values in STEM students in the higher education context.

#### 3.3.1 STEM students in the innovation model

STEM students begin their higher education in this discipline because it is challenging. They are responsible for working hard and becoming involved in the STEM environment provided by their university. They should also cooperate with their peers and professors in building a suitable and inclusive environment where less advantaged students can have vicarious mastery experiences while valuing deep approaches to learning [35]. Students are ultimately responsible for seeking help when facing obstacles, including overcoming the shortcomings of their previous basic education. Students should not see themselves as consumers of a product but as privileged members of society who are building scientific capital that will benefit them as individuals and professionals who can develop the foundations for innovation. They should hold professors and universities accountable for providing high-quality education. A summary of the goals, values, and behaviors that students should develop in STEM education is shown in Fig. 6.

#### 3.3.2 The STEM teacher in the innovation model

A STEM teacher is the first role model a student encounters in higher education. Teachers must convey the importance, beauty, and joy of STEM disciplines, encourage students to participate in innovative practices and see themselves as members of a society that produces and applies knowledge. They should ensure that they offer students a safe and comfortable environment. They are responsible for providing high-quality education that involves performing scientific practices, fostering technoscientific values and innovative practices, and challenging students to give their best. Students should be assisted in finding alternatives and solutions when seeking help. A summary of the goals, values, and behaviors that STEM professors should master is shown in Fig. 6.

#### 3.3.3 The education institution in the innovation model

STEM education occurs in this setting. Given its ability to influence student values, it plays a vital role. This institution provides an adequate and accessible framework for STEM education. This includes but is not limited to providing facilities and resources for technoscientific practices. The institution must ensure that students and teachers have a safe space to learn and teach while being promptly protected from harassment and discrimination. It must also provide counseling and tutoring for struggling students, ensure that teachers are equipped to perform to their best, and hold students and professors equally accountable. Educational institutions should also display goals, values, and behaviors, as shown in Fig. 6.

#### 3.3.4 The government/state in the innovation model

The government has set regulations that direct STEM education, as it is responsible for establishing policies that favor research, innovation, and commercialization [21]. However, its role is broader than providing curricular content or quality assurance. Authorities should ensure that higher education institutions are accessible to every student, that students carry the necessary academic and personal skills when reaching higher education, and that inequities are minimized and do not become obstacles to students. The government must see students as future innovators who will bring goods to society, the economy, politics, and the world. An effective STEM education policy is an investment in the future. The goals, values, and behaviors that are important for governments are summarized in Fig. 6.

This study analyzed the literature to propose a new model (Fig. 6). Although a value-based approach to education could sound innovative to many people, the results may only represent a fraction of the total picture. In this review, social values were emphasized in the literature; however, given that the search queries focused on values, it is possible that other studies examining curricular content and performance evaluations were excluded. This systematic review complements other previous systematic reviews [33], showing that students who prioritize content mastery and innovative thinking rather than course performance and who see themselves as students instead of consumers tend to perform better and have greater self-efficacy when studying STEM.

This is the first systematic review and ethical meta-analysis to examine the values that have emerged from the literature. This article reflects on some of the important values that appear in the STEM education organizational culture. This study is original, as it weaves several ideas, opinions, and theories presented in different papers and hunts for values that are not explicitly showcased. This allowed us to build a model based on the value systems considered relevant in the literature, those that still require strengthening, and those that we believe should be included.

While no other studies have investigated the values of STEM education organizational culture, this study is limited because it only examines the values arising in the STEM education literature. While these values are considered necessary by STEM education researchers and are part of the STEM education organizational culture, they are not necessarily the same as found in practice by STEM students, professors, school administrators, and the government.

STEM education researchers can establish part of the agenda of priorities in STEM education organizational cultures. However, according to the competing values model [22], every party in the organization places its values on the table. Cultural values result from the tension between all goals, ends, values, and behaviors of every stakeholder involved. Furthermore, while the value systems in STEM education do not tend to change significantly, the relationship between them and their hierarchies is dynamic in terms of time and region. Therefore, the results of this study may not apply to the future decade and may be limited to only developed nations.

Concretely speaking, and based on the results of this paper, we recommend that policy-makers and STEM educators first visualize STEM education as a system in which four stakeholders interact—students, instructors/teachers, educational institutions, and the government/state. This facilitates identifying each party's goals, ends, and values. A second step involves establishing the value systems for each party and then proposing their goals and values.

In Fig. 6, we propose several goals and values, but these may vary depending on the context in which STEM education occurs. With these findings in mind, the third step involves assigning each party-specific responsibility, which includes the innovation component of STEM. This will build the foundation for strategically developing an action plan for each stakeholder.

It is important to mention that for top-down educational policy, it may be appropriate to include the governance component in the model (government/state). For local educational innovations, the governance and even institutional components of the model may be fixed. Finally, it is important to establish a value-based follow-up strategy to evaluate and adapt the innovation model so that it evolves along with the current needs of the four stakeholders.

## 4 Conclusions

This is the first research paper that performs an ethical meta-analysis of the current literature on STEM higher education, outlining the values that emerge within this field and proposing an innovation model. This article contributes to the knowledge base of STEM education by offering a novel, value-based perspective on current issues in the discipline. A value-based approach to emerging issues can assist in proposing new solutions to problems and provide a more comprehensive array of indicators for evaluating policies and educational interventions/innovations.

This study aims to identify the emerging value systems in the most recent literature on STEM education, highlight the leading topics of discussion and research that still require more discussion, and determine the main actors in STEM education. It also proposes a cross-functional model that outlines the responsibilities of each party. Values have not been explicitly studied in the current STEM education literature, and innovation-directed STEM education organizational culture has only been tangentially addressed. For this reason, we undertook a “value-hunting” approach. The current literature underscores the social value of STEM education. Social values emerge when discussing equal access to STEM education, the recognition and prestige of the scientist, cooperation between students, and cooperation between students and the professor to build an epistemic background and when discussing the consequences of science.

Four STEM stakeholders were identified in the review (see Fig. 6): students, teachers, higher education institutions, and the government. The literature focuses on the utilitarian ethical approach by emphasizing the importance of conveying the usefulness of science. Very few studies discuss the duties and virtues of each stakeholder. While the literature shows the utility of course content in fostering student commitment (economic values), it neglects the relationship between other value systems and the responsibilities of each stakeholder.

This approach does not consider the complexity of issues involving multiple parties. Each of the previously mentioned stakeholders must focus on their manifold responsibilities and not be burdened by the responsibilities of the other parties. For example, while inequities in scientific capital distribution are essential issues to consider so that STEM teachers do not replicate oppressive structures in class, course instructors cannot completely address these problems independently. The role of professors in tackling these social issues in the classroom requires more comprehensive and realistic exploration. Moreover, unprivileged students may require support that neither STEM teachers nor educational institutions can provide.

We propose a values-based model that identifies pending STEM education ethical issues (SEEIs) that can help guide decision-making by underscoring what is vital to STEM students, STEM teachers, higher education institutions, and the government. The model establishes integral responsibilities so that each of the stakeholders can contribute to creating a local STEM *ethos*. These responsibilities are based on core values deemed necessary in the literature, values that can still be bolstered to improve STEM educational practices, and values that still need to be strengthened and cultivated.

STEM students need to commit enthusiastically to the scientific nature of STEM disciplines while seeking help and support, if needed. STEM professors/instructors must ensure that the classroom is a safe and comfortable space for students and serve as role models that challenge STEM students to achieve more. Higher education institutions must provide adequate infrastructure so that STEM professor–STEM student relationships can flourish productively. Finally, the government should establish a context in which higher education institutions should work to harness innovation. It is essential to emphasize that this model is meant to establish a direction in which studying and teaching STEM can be performed meaningfully because sharing and distributing expectations, responsibilities, and commitments between stakeholders will help them work toward a common purpose. This will bring about virtuous teaching practices that pave the way for innovation as an end to a STEM *ethos*. Helping each party assume responsibility for developing STEM education is the only way to foster technoscientific values in the future.

One of the most significant contributions of this study is that it establishes the foundation for an innovative culture in STEM education. In this study, we conceive of innovation culture as new future-oriented ideas that foster and strengthen several behaviors and attitudes, such as openness to change, risk-taking, tolerance to mistakes, experimental work, creativity, and the search for truth. These behaviors go beyond course performance and create a value-directed (virtuous) environment where students act freely and cooperate with different parties to create new, untold opportunities to solve problems and serve their communities and societies.

Our findings underscore the salient features of a values-based innovation culture amalgamating elements from different organizational cultures (i.e., adhocracy, clan, commercial, or hierarchical cultures). Each type of culture favors a set of value systems that ensures success. For example, an adhocracy culture favors dynamism and creativity, whereas loyalty, tradition, and teamwork are fostered in clan cultures. The model presented in this study goes beyond the social values currently nurtured in STEM education research. Our model requires the multicultural coexistence of values, highlighting the systems that should be given priority depending on the context.

The clan culture values that promote maintaining the *status quo* work well when quick reactions are required (i.e., in an emergency); however, adhocracy and commercial culture values are important when dynamism, creativity, and profits are favored. Leaders should demonstrate wisdom and prudence when setting the values at stake in each situation. The proposed model allows us to put this recommendation into practice by promoting the idea that every stakeholder should be able to achieve their STEM educational goals. This is closely related to the ethical use of science and technology to improve society. The main goal in STEM higher education should be to plant in students the idea that value dynamism is the catalyst for comprehensive and integral technoscientific innovation.

## Data availability

Data included in article/supp. material/referenced in article. Coding information on Atlas.ti is available from the first author upon request.

## Funding

This research received no specific grant from funding agencies in the public, commercial, or not-for-profit sectors.

## Ethical statement

Not Applicable.

## Consent statement

Not Applicable.

## CRediT authorship contribution statement

**Fernand Vedrenne-Gutiérrez:** Writing – review & editing, Writing – original draft, Methodology, Investigation, Formal analysis, Data curation, Conceptualization. **Carolina del Carmen López-Suero:** Supervision, Resources, Investigation. **Adalberto De Hoyos-Bermea:** Validation, Resources, Methodology, Investigation. **Lorena Patricia Mora-Flores:** Investigation, Formal analysis. **Daniela Monroy-Fraustro:** Investigation, Formal analysis. **María Fernanda Orozco-Castillo:** Investigation, Formal analysis. **José Francisco Martínez-Velasco:** Validation, Supervision, Investigation. **Myriam M. Altamirano-Bustamante:** Writing – review & editing, Validation, Supervision, Resources, Project administration, Methodology, Investigation, Formal analysis, Conceptualization.

## Declaration of competing interest

The authors declare that they have no known competing financial interests or personal relationships that could have appeared to influence the work reported in this paper.
